This article has been retracted.

# Radical Covalent Organic Frameworks Associated with Liquid Na‐K toward Dendrite‐Free Alkali Metal Anodes

**DOI:** 10.1002/advs.202203058

**Published:** 2022-07-21

**Authors:** Jianyi Wang, Menghui Chen, Zicong Lu, Zhida Chen, Liping Si

**Affiliations:** ^1^ School of Materials Science and Hydrogen Energy Foshan University Foshan 528000 P. R. China; ^2^ Institute for Sustainable Energy/College of Sciences Shanghai University Shanghai 200444 P. R. China

**Keywords:** alkali metal batteries, covalent organic frameworks, Na‐K alloys, self‐healing, stable ability

## Abstract

Liquid sodium‐potassium (Na‐K) alloy has the characteristics of high abundance, low redox potential, high capacity, and no dendrites, which has become an ideal alternative material for potassium/sodium metal anodes. However, the high surface tension of liquid sodium potassium alloy at room temperature makes it inconvenient in practical use. Here, the Na‐K as reducing agent treats with hydrazone linkages of covalent organic frameworks (COFs) and obtain the carbon‐oxygen radical COFs (COR‐Tf‐DHzDM‐COFs). The preparation method solves the problems that the preparation process of the traditional Na‐K composite anode is complex and has high cost. The structures of the COR‐Tf‐DHzDM‐COFs are characterized by X‐ray diffraction （XRD), fourier transform infrared (FT‐IR), electron paramagnetic resonance (EPR), and solid‐state NMR measurements. It is the first time that carbon‐oxygen radical COFs from bulk COFs are constructed by one‐step method and the operation is flexible, convenient, and high rate of quality, which is suitable for big production and widely used. The cycle stability of the composite Na‐K anode is improved, which provides a new idea for the design of high‐performance liquid metal anode.

## Graphical abstract

Radical COFs realized by the incorporation of Na‐K alloy are applied as non‐Newtonian viscous liquid anode. Due to the high surface tension and good structural stability, the new non‐Newtonian fluid COR‐Tf‐DHzDM‐COFs@NaK exhibits excellent electrochemical performance.

## 1 Introduction

With the wide application of portable electronic equipment and electric vehicles, higher requirements are put forward for high energy density batteries.^[^ ^1^ ^]^ Although metal electrodes have high energy density, for most alkali metal anodes, uneven alkali ion deposition can lead to dendrite formation and hinder the further application of rechargeable alkali metal‐based batteries.^[^ ^2^ ^]^ Among them, the liquid metal anode has deformation and self‐healing properties, which can slow down the volume change caused by metal dendrite growth during the cycle.^[^ ^3^ ^]^ For example, a new flexible lithium‐ion battery anode was developed by room temperature gallium‐based liquid metal and two‐dimensional material of MXene.^[^ ^4^ ^]^ As for the more economical alkali metal of sodium and potassium would be more versatile.^[^ ^3a^ ^]^ However, obtaining common metals in liquid phase usually requires high temperature operation, which will bring safety problems and additional energy consumption. Unlike ordinary metals, sodium potassium (Na‐K) alloys can be stable in liquid phase at room temperature.^[^ ^5^ ^]^ These excellent properties make Na‐K alloy an excellent anode material in alkali metal‐based batteries, and alleviate the formation of dendrites and short circuit.

Due to advantage of radical organic material tends to have a highly active and fast reaction kinetics and lack of the high active of free radical middle substance is unstable due to its unpaired electrons and reaction with other activity factor.^[^ ^6^ ^]^ Therefore, regulating the stability of radical intermediates by grafting the radical monomer to covalent organic frameworks (COFs) is one of the ways to optimize the performance.^[^ ^1^, ^7^ ^]^ The previous of study pointed out that nitrogen‐oxygen/carbon‐oxygen/carbon/nitrogen radical COFs for catalyst^[^ ^8^ ^]^ and electrode^[^ ^6^, ^9^ ^]^ have a highly active and fast reaction kinetics, which is helpful in rate of reaction. The spatial effect of unpaired electrons can be de‐localized by ionization and *π*–*π* conjugate interaction, and the self‐exchange behavior of intermolecular electrons can be restricted. Rigid big rings are often used to regulate the stability of radical intermediates, which can inhibit dissolution in electrolyte, transport charge by *π* conjugated frameworks and transport ions by a large number of nanoporous.^[^ ^10^ ^]^ However, the current synthesis of radical‐based COFs requires linking radical units, which increases the threshold. In addition, the preparation process of the traditional direct synthetic radical COFs are complex and has high cost, which greatly limits their application.^[^ ^8^, ^9^, ^11^ ^]^ the radical monomer is unstable and complex synthesis process, which hinders the research work to go deeper. Hence, here reports a special method that used a liquid alkali metal (Na‐K alloy) reducing agent, the successfully in situ construction of carbon‐oxygen radical COFs (COR‐Tf‐DHzDM‐COFs) in bulk quantities using a simple and cheap process. The whole preparation process (mixing and filtering) is simple and feasible, does not need special apparatuses, has low cost and is suitable for mass production and promotion. Significantly, the raw COFs of Tf‐DHzDM‐COFs (1,3,5‐Benzenetricarboxaldehyde and 2,5‐dis‐ubstituted terephthalohydrazide (DHzDM)) don't need a higher temperatures and long reaction time (**Figure** **1**). Through the Electron Paramagnetic Resonance (EPR) spectra, the paper has described the radical of COR‐Tf‐DHzDM‐COFs, the peaks of the functional characteristic showed up, proving that the paper has synthesized the target products. The chemical composition and stability characterizations of COR‐Tf‐DHzDM‐COFs are studied and discussed. In addition, the COR‐Tf‐DHzDM‐COFs combine with Na‐K alloy has lots of advantage acting as the electrode material, and has huge application potential. With the controllable pore structure, abundant functional radical organic groups and good mechanical properties of COR‐Tf‐DHzDM‐COFs, Na‐K can quickly diffuse in COR‐Tf‐DHzDM‐COFs, so as to realize the liquid metal anode easy to use at room temperature. In addition, due to the excellent dynamic properties of liquid Na‐K alloy and the excellent electron/ion transport properties of COR‐Tf‐DHzDM‐COFs, COR‐Tf‐DHzDM‐COFs@Na‐K composite anode can not only effectively inhibit dendrite, but also exhibit excellent cycle stability. This work provides a new direction for the development of high‐energy alkali metal batteries and an important background for the development of liquid metal anodes.

**Figure 1:** a) Design and synthesis of COR‐Tf‐DHzDM‐COFs. The reduction reaction occurs in one step and form an oxygen vacancy defects (the digital video show the process in supporting material). b) The synthesized routes of the COR‐Tf‐DHzDM‐COFs. c) Schematic illustration of fabrication process of Tf‐DHzDM‐COFs@Na‐K anode and preparation of non‐Newtonian flow Tf‐DHzDM‐COFs@Na‐K composites and composite anode at room temperature for dendrite‐free metal battery.

## 2 Results and Discussion

The synthesized routes of the COR‐Tf‐DHzDM‐COFs is shown in Figure 1b. Tf‐DHzDM‐COFs was prepared through Schiff base reaction according to the literature,^[^ ^12^ ^]^ and the COR‐Tf‐DHzDM‐COFs was prepared by the Na‐K alloy treatment. Tf‐DHzDM‐COFs is a white solid, which gradually changes from white to blue when treated. The process of color change is due to the emergence of radical organic groups in Tf‐DHzDM‐COFs, which forms a new band and shows blue. The progress of synthesis of COR‐Tf‐DHzDM‐COFs@Na‐K composites is shown in Figure 1c. Firstly, liquid Na‐K alloy is formed by mixing and stirring solid K metal and Na metal (mass ratio 3:1) at room temperature (25 °C). Na‐K alloy and COR‐Tf‐DHzDM‐COFs are then mixed and stirred for several minutes, so that the COR‐Tf‐DHzDM‐COFs particles are composite with a uniform liquid alloy and can be prepared into a non‐Newtonian viscous liquid (COR‐Tf‐DHzDM‐COFs@Na‐K). In order to intuitively characterize the defects types in samples prepared under different treatment conditions, solid EPR spectra were carried out. **Figure** **2**a shows the EPR spectra of raw materials Tf‐DHzDM‐COFs and COR‐Tf‐DHzDM‐COFs. It can be seen that in the EPR spectra, after Na‐K alloy treatment there is an obvious symmetrical signal peak at magnetic field = 322.3 mT, while no such a signal has been observed for the raw material. The EPR peak defines a carbon‐oxygen radical signal, indicating that form a great of quantities carbon‐oxygen radical in sample.^[^ ^13^ ^]^ The existence of radical confirms the abundant of oxygen vacancies in COR‐Tf‐DHzDM‐COFs. Therefore, according to the EPR results, we can confirm that the Na‐K alloy treatment promotes the generation of carbon‐oxygen radical in Tf‐DHzDM‐COFs.

**Figure 2:** Morphological and structural characterizations of Tf‐DHzDM‐COFs. a) EPR curves, b) XRD patterns, c,d) HRTEM image of Tf‐DHzDM‐COFs and COR‐Tf‐DHzDM‐COFs, respectively. e,f) HRTEM image of Tf‐DHzDM‐COFs and COR‐Tf‐DHzDM‐COFs, respectively.

The crystal structure of the COR‐Tf‐DHzDM‐COFs was further tested by X‐ray powder diffraction (XRD) instrument (Figure 2b). All diffraction peaks can be well assigned to the Tf‐DHzDM‐COFs,^[^ ^12^ ^]^ indicating that there is no impurity generated, and the COR‐Tf‐DHzDM‐COFs has a high crystallinity. The result suggested that Na‐K alloy treatment is an efficient and convenient way to prepare carbon‐oxygen radical in the COFs. Beside, during the reduction reaction, Na‐K alloys consumed the oxygen element in the Tf‐DHzDM‐COFs and the oxygen was finally oxidized to the corresponding oxides (Na_x_‐O‐C‐ and K_x_‐O‐C‐), which can be removed from the crystalline structure through sufficient washed with water. This method is suitable for large‐scale production of carbon‐oxygen radical COFs materials. Depending on all above studies and experiments, we can conclude that using Na‐K alloy treatment rules in carbon‐oxygen radical synthesis is viable. More than anything, the proposed method can also be applied to similar tasks.

In order to investigation and study the inner structure changes of the Tf‐DHzDM‐COFs caused by reduction of Na‐K alloy. The difference was also characterized by transmission electron microscopy (TEM) and scanning electron microscopy (SEM), as shown in Figure 2c–f, respectively. Compared with the Tf‐DHzDM‐COFs, the treated COFs shows many complex lattice stripes, which are the amorphous phenomenon caused by the carbon‐oxygen radical. The amorphous areas shown in the blue line, which indicates that the absence of oxygen in COR‐Tf‐DHzDM‐COFs caused partial lattice destruction. While the crystal lattice fringes could be clearly seen in the Tf‐DHzDM‐COFs, which had a good long‐term orderly arrangement, and there was no disordered area in the internal structure of Tf‐DHzDM‐COFs. From the pore size distribution of the samples before and after mixture with Na‐K (Figure S1, Supporting Information), it was not difficult to find that the pore volume also decreased when the specific surface area decreased, but the pore size remained unchanged. This is because carbon‐oxygen radicals are mainly present in the internal structure of the Tf‐DHzDM‐COFs. Comprehensive consideration Figure 2 and Figure S1 (Supporting Information), all suggest that the Tf‐DHzDM‐COFs with carbon‐oxygen radical was successfully obtained. In addition, the morphology has no obvious changes after the Na‐K alloy treatment. With all of these changes and non‐changes together, we do believe that the specialists working in developing the carbon‐oxygen radical in polymeric crystal structure will change the electronic structure of COFs, which lays a good foundation for the future developing trend of high‐performance carbon‐oxygen radical COFs used in all aspect of Chemistry and Materials.^[^ ^14^ ^]^ In addiction, the electrochemical performance of half‐cell with COFs and the composites anode was tested. CV test showed that a Na+/K+ intercalation potential of 0.5–1 V (3M KFSI/DME, a half‐cell of potassium‐ion battery (Figure S2, Supporting Information). It shows that the method of regulating oxygen vacancies in COFs mainly depends on the introduction of alkali metal ions with different electronic effects.

A better understanding of the effects of Na‐K alloy treatment on the presence form of O element in COR‐Tf‐DHzDM‐COFs at molecular levels is performed by Fourier Transform Infrared Spectroscopy (FT‐IR, **Figure** **3**a) and solid state nuclear magnetic spectra (NMR, Figure 3b). Both the FT‐IR and NMR spectra remained basically unchanged after treatment, indicating that the frame structure was maintained.^[^ ^15^ ^]^ There are slight changes for the carbonyl group both in the FT‐IR and NMR spectra. Close analysis of the FT‐IR spectra, the peak at 1305–1200 cm^−1^ was flattened compared to the raw material; and in the NMR spectra the peak at 127.45 ppm was also overlapped by the neighboring peak. All this indicating the occurrence of the carbon‐oxygen radical, which weakens the original signal.

**Figure 3:** Representative a) FT‐IR spectra, b) ^13^C CP‐MAS solid‐state NMR spectra, c) O1s, and d) K 2p‐C1s XPS spectra of Tf‐DHzDM‐COFs and COR‐Tf‐DHzDM‐COFs.

Furthermore, XPS experiment was used to characterize the O, C element of COR‐Tf‐DHzDM‐COFs and Tf‐DHzDM‐COFs, and the fitting spectrum obtained is shown in Figure 3c,d. The O1s spectrum of Tf‐DHzDM‐COFs can be generally divided into two peaks: the binding energy of 531.5 eV (O1) can be ascribed to oxygen vacancy defect in the lattice; the other binding energy of 533.5 eV (O2) can be ascribed to surface adsorbed oxygen.^[^ ^16^ ^]^ Therefore, we obtained high fitting degree by peaking O1S spectra of the Tf‐DHzDM‐COFs. There is a certain proportion of carbon‐oxygen radical in both the Tf‐DHzDM‐COFs and the COR‐Tf‐DHzDM‐COFs. Because all crystals are not perfect, there is a certain concentration of intrinsic defects. For Tf‐DHzDM‐COFs, the formation energy of carbon‐oxygen radical in the intrinsic defect is the lowest, so the Tf‐DHzDM‐COFs inevitably has a small amount of oxygen vacancy. Meanwhile, the K 2p spectra suggested that there are no K elements (binding energy: 298–290 eV) in the COR‐Tf‐DHzDM‐COFs, indicating that all the alkali‐metal had been removed.^[^ ^17^ ^]^ Furthermore, Figure S3 (Supporting Information) shows the N1s binding energy of COR‐Tf‐DHzDM‐COFs and Tf‐DHzDM‐COFs is 401.0 and 401.3 eV, respectively. After the Na‐K alloy treated, the N1s binding energy of COR‐Tf‐DHzDM‐COFs shifts to lower binding energy,^[^ ^18^ ^]^ indicating that the chemical environment around N element changes. Obliviously, it can be seen that the proportion of oxygen vacancy in the COR‐Tf‐DHzDM‐COFs is significantly higher than that of Tf‐DHzDM‐COFs, indicating that the carbon‐oxygen radical concentration increases. It can be understood as a short time after the treatment of Na‐K alloy reducing, some position of oxygen can under strong reduction and leaving the original position left oxygen vacancy, which also verified from the EPR. The results further prove that the COR‐Tf‐DHzDM‐COFs is a kind of porous crystallinity material with carbon‐oxygen radical.

All this above experiment suggested that treated with the Na‐K alloy, carbon‐oxygen radical was introduced into the pristine COFs structure without destroy the frameworks. The effectiveness of carbon‐oxygen radical COFs will focus on some results that would be stable in variety environment. The resistance of the COR‐Tf‐DHzDM‐COFs with acid/alkali solution and thermal stability was also tested and discussed. Firstly, the COR‐Tf‐DHzDM‐COFs was immersed in 20 mL 1 m sulfuric acid and 1 m hydrochloric acid, for 24 h, and then the solid was filtered and dried. The X‐ray powder diffraction (XRD) was used for analysis and comparison the anti‐acidity of carbon‐oxygen radical in COR‐Tf‐DHzDM‐COFs (Figure S4, Supporting Information), which showed that carbon‐oxygen radical has good stability in 1 m sulfuric acid due to stable framework of COFs, which can provide rigidity structure support for the highly active radical. For another acid of 1 m hydrochloric acid, the results show the COR‐Tf‐DHzDM‐COFs still have a slightly peaks. It is worth noting that COR‐Tf‐DHzDM‐COFs is stable when dissolved in higher levels of 2 m hydrochloric acid and strongly basic solutions of 1 m potassium hydroxide. The EPR was used for analysis and comparison the anti‐acidity of carbon‐oxygen radical in COR‐Tf‐DHzDM‐COFs (Figure S5, Supporting Information). Figure S5a (Supporting Information) shows that carbon‐oxygen radical has good stability in 1 m sulfuric acid due to stable framework of COFs, which can provide rigidity structure support for the highly active radical. For another acid of 1 m hydrochloric acid, the results show the COR‐Tf‐DHzDM‐COFs still have a slightly peaks (Figure S5b, Supporting Information).

To further investigate the thermal stability of COR‐Tf‐DHzDM‐COFs, we tested their thermal stability using a thermogravimetric analyzer (Figure S6, Supporting Information). Prior to testing the thermal stability, the thermogravimetric curve of COR‐Tf‐DHzDM‐COFs showed that ≈44.5% of the massless at 30–150 °C could be instructions the weight loss of the solvent molecules in the internal structure of COR‐Tf‐DHzDM‐COFs. The COR‐Tf‐DHzDM‐COFs stabilized to about 370 °C, and then the COR‐Tf‐DHzDM‐COFs frame began to collapse and decompose, causing a sharp drop in the thermogravimetric curve. The samples exhibited high thermal stability with Tf‐DHzDM‐COFs.

Tf‐DHzDM‐COFs on the structure of the Tf‐DHzDM‐COFs with Na‐K alloy could provide a new way to modify the electrochemical property for liquid alkali metal batteries. The composite anode was formed by placing it in a Cu foam current collector and applied to the battery test.

The symmetrical cells were used to evaluate the electrochemical properties of COR‐Tf‐DHzDM‐COFs@Na‐K and pure K electrodes (**Figure** **4**a,c). Obviously, COR‐Tf‐DHzDM‐COFs@Na‐K@Cu foam shows smaller voltage fluctuations and longer cycle lives than K electrodes. The full cell is assembled with COR‐Tf‐DHzDM‐COFs@Na‐K@Cu foam and K as the anode and Prussium potassium blue (KPB) as the positive electrode (Figure 4b,d). COR‐Tf‐DHzDM‐COFs@Na‐K@Cu foam also showed stronger electrochemical performance, but the role of COR‐Tf‐DHzDM‐COFs in this process remains to be further studied. The polarization voltage of the composite anode is only 340 mV, and it can cycle stably for 200 h. In order to reflect the influence of the anode material on the electrochemical performance of the whole battery, we used sodium vanadium phosphate (NVP) with a stable structure and a voltage platform of about 3.4 V as the cathode material, which can stable cycle more than 100 times without obvious capacity attenuation, and maintain the Coulomb efficiency above 99% in the whole cycle process (Figure 4e,f). It should be noted that there are few K^+^ involved in the electrochemical reaction, which will not affect the liquid state of Na‐K changes after K stripping. Similar reference also shows excellent performance with Na‐K alloy anode.^[^ ^5^, ^19^ ^]^

**Figure 4:** Battery stability measurement. Symmetric cell stability in potassium metal anodes (KMBs) a) COR‐Tf‐DHzDM‐COFs@Na‐K, and c) pure K metals (current density: 0.5 mA cm^−2^). Full cell cycling performances of COR‐Tf‐DHzDM‐COFs@Na‐K@Cu foam//KPB b,d) pure K//KPB metals after activation (current density: 0.2 A g^−1^). e) Symmetric cell (current density: 1 mA cm^−2^) and f) Full cell (current density: 0.2 A g^−1^) cycling performances of COR‐Tf‐DHzDM‐COFs@Na‐K@Cu foam in sodium metal anodes (SMBs).

According to the EPR pattern of the COR‐Tf‐DHzDM‐COFs after cycles (Scrape the powder off from anode and wash it by DMC, Figure S7, Supporting Information), there is still a large amount of carbon‐oxygen radical in the powder of COR‐Tf‐DHzDM‐COFs, which fully indicates that the COR‐Tf‐DHzDM‐COFs ‐based composite anode can be the potential composite anode material for alkali metal anode.

The battery still shows excellent rate performance and cycle performance at low temperature (**Figure** **5**). The composite electrode can cycled at 1 mA cm^−2^ for more than 60 h at −20 °C. Using the composite anode, A full battery with NVP and KPB as the cathode and COR‐Tf‐DHzDM‐COFs@Na‐K@Cu foam has a high capacity of 67% after 100 cycles of 0.2 A g^−1^ at −20 °C. Over a 100‐cycle recharge test, performance remained acceptable. In the future, other high‐performance alkaline batteries are expected to be developed. Based on the above analysis and indicate that COR‐Tf‐DHzDM‐COFs modified Na‐K alloy anode can effectively improve the cycle life of alkali metal battery.

**Figure 5:** a) Symmetric cell (current density: 0.5 mA cm^−2^) and b) Full cell (current density: 0.2 A g^−1^) cycling performances of COR‐Tf‐DHzDM‐COFs@Na‐K@Cu foam in KMBs at −20 °C. c) Symmetric cell (current density: 1 mA cm^−2^) and d) Full cell (current density: 0.2 A g^−1^) performances of COR‐Tf‐DHzDM‐COFs@Na‐K@Cu foam in SMBs at −20 °C.

## 3 Conclusion

Radical is an important branch in organic materials, which plays an important role in improving the performance of materials. In this paper, a simple and efficient method of producing carbon‐oxygen radical in COFs assisted by Na‐K alloy is innovatively proposed. Taking Tf‐DHzDM‐COFs as the research subject, the mechanism of strong reducing action to produce carbon‐oxygen radical and its effect on material properties and reasons were explored. The general applicability of the method of producing carbon‐oxygen radical by Na‐K liquid metal assisted treatment was investigated with various COFs. In addition, through the study and characterization of the composite formed by mechanical mixing of Tf‐DHzDM‐COFs and Na‐K alloy, it is confirmed that the composite anode of Na‐K alloy can inhibit the dendrite growth and thus show stable circulation at both ultra‐low temperature (−20 °C) and room temperature. Therefore, it can be considered that the COR‐Tf‐DHzDM‐COFs studied in this paper brings new possibilities for defect engineering to improve material properties, and this work has universal significance in many research fields.

## Conflict of Interest

The authors declare no conflict of interest.

## Supporting information

Supporting Information

Supplemental Video 1

## Data Availability

The data that support the findings of this study are available from the corresponding author upon reasonable request.
